RETRACTED

# Pemetrexed for Recurrent Primary Central Nervous System Lymphoma in the Elderly: Results of a Retrospective Study

**DOI:** 10.1155/2022/8963547

**Published:** 2022-03-29

**Authors:** Jing Xiao, Shishu Wang, Bing Xu, Lisha Yu, Yan Han

**Affiliations:** ^1^Department of Hematology, Yantaishan Hospital, Yantai 264000, China; ^2^Department of Hematology, The Affiliated Qingdao Central Hospital of Qingdao University, The Second Affiliated Hospital of Medical College of Qingdao University, Qingdao 266042, China; ^3^Department of Neurology (I), The Affiliated Qingdao Central Hospital of Qingdao University, The Second Affiliated Hospital of Medical College of Qingdao University, Qingdao 266042, China; ^4^Department of Traditional Chinese Medicine, Qingdao Eighth People's Hospital, Qingdao 266000, China; ^5^Department of Gastroenterology, The Second Affiliated Hospital of Shandong University of Traditional Chinese Medicine, Jinan 250001, China

## Abstract

**Aim:**

Primary central nervous system lymphoma (PCNSL) is an aggressive, destructive, and rapidly progressive malignant brain tumor. Although aggressive therapies were studied trying to increase the median survival of PCNSL, the high relapse rate of PCNSL is still a big problem for the oncology medicine. A retrospective study was made to evaluate the efficacy and safety of pemetrexed in the treatment of patients with recurrent PCNSL.

**Methods:**

Twenty-three confirmed recurrent PCNSL patients were selected during April 2012 and August 2016. Dexamethasone, B_12_, and folic acid were used to produce the toxicity related to pemetrexed. The patients were intravenously given pemetrexed (900 mg/m^2^) every three weeks for 6 weeks.

**Results:**

After the treatment, 7 patients were in complete remission, 6 patients in partial remission, 4 patients in stable condition, and 6 patients in progression. There were 56.5% and 73.9% in the overall response rate and the disease control rate, respectively. The median overall survival (OS) was 6.6 months (95% CI, 4.6–8.6).

**Conclusion:**

This study has been the first time to evaluate the safety and effectiveness of pemetrexed on elderly recurrent PCNSL patients. Results demonstrate that using high-dose pemetrexed might be a feasible and effective treatment for recurrent PCNSL in the elderly, and clinical trials should be conducted to further confirm it.

## 1. Introduction

Primary central nervous system lymphoma (PCNSL) is an aggressive, destructive, and rapidly progressive malignant brain tumor. Although the median survival for high-methotrexate-based active therapy is about 30–50 months, the high relapse rate of PCNSL is still a big problem in oncology [1–6]. Studies indicated that the survival time of recurrent PCNSL is between 2 and 14 months, and it was worse in the elderly [7, 8]. Particularly, compared with young PCNSL patients, the elderly PCNSL patients were more likely to relapse early after the initial treatment. However, there is no standard salvage treatment for recurrent PCNSL in the young and elderly patients [9–12]. The research focus of PCNSL has always been to explore effective treatment methods.

RETRACTED

Due to the poor prognosis of elderly patients with recurrent PCNSL, novel drugs need to be evaluated. Pemetrexed is a typical antitumor drug, which is a folic acid antagonist such as methotrexate. However, pemetrexed has the superiority of multiple targets than one site in folic acid metabolism, which can kill tumors efficiently by infiltrating into the central nervous system [13]. Several studies have evaluated the safety and efficacy of pemetrexed in the treatment of recurrent PCNSL, but substantive research is still scarce [13–15]. Moreover, these studies were only focused on the general population lacking specific people. In this study, the elderly recurrent patients were focused to assessing the efficacy and safety of pemetrexed on recurrent PCNSL.

## 2. Methods

### 2.1. General Information

The retrospective study was performed at the Yantaishan Hospital and was approved by the ethical review board of the hospital. The medical records and imaging data of patients with recurrent PCNSL treated with pemetrexed from April 2012 and August 2016.

#### 2.1.1. Inclusion Criteria

All elderly patients with PCNSL were progressed during the first-line chemotherapy and/or radiotherapy, or recrudesced after initial successful treatment. All patients had radiographically measurable intracranial disease, in which the tumor was detectable in two dimensions (at least 1 cm × 1 cm) by contrast-enhanced magnetic resonance imaging (MRI) with Crabuak. Chemotherapy was the first choice after the diagnosis. However, all patients with recurrent PCNSL were received radiotherapy, if the disease progression was not controlled by chemotherapy. All patients were over 65 years of age, and initial biopsies proved negative for immune system disease. Patients' life expectancy was greater than 3 months and Karnofsky performance status (KPS) was ≥50. Also, patients need to have adequate blood, kidney, and liver function.

### 2.2. Therapeutic Schedule

Pemetrexed at 900 mg/m^2^ were administered every 3 weeks of a 6-week cycle. To minimize pemetrexed-related toxicities, 0.4 mg folic acid was given daily at the first dose of pemetrexed 1 week before and 3 weeks after the treatment. Considering the prevention of pemetrexed-induced rashes, 4 mg dexamethasone was given twice daily during one day before and one day after the treatment. 1 mg vitamin B_12_ was also injected intramuscularly in two consecutive periods, including 2 weeks before the first use of pemetrexed and at 9-week intervals during treatment. Pemetrexed treatment was remained as long as without evidence of complete response, intolerable side effects, or tumor progression. Additionally, mannitol (20%) was injected intravenously with a high rate at each time before and after the chemotherapy to increase blood-brain barrier permeability.

RETRACTED

### 2.3. Evaluation Methods

Baseline evaluation standard and response criteria were used according to the 2005 PCNSL neuroradiographic response criteria of the international lymphoma working group, including four levels for response. In order to evaluate the efficacy of the pemetrexed treatment in elderly PCNSL, the disease control rate and overall response rate were calculated as the sum of PR and CR, and the sum of PR, CR, and SD, respectively.

According to National Cancer Institute Common Terminology Criteria for Adverse Events (version 4.0), the side effects were assessed as 0–v grades and toxicity was classified as mild (level 1), moderate (level 2), severe (level 3), life-threatening (level 4), or death (level 5). Patients were removed if they had PD, developed unacceptable toxicity, or refusal or did not comply with protocol requirements.

### 2.4. Statistical Analysis

The time of OS and progression-free survival were calculated for each patient. The Kaplan–Meier method was used to calculate the survival curve, and SPSS 16.0 was performed for all statistics.

## 3. Results

### 3.1. Patient Characteristics

Among twenty-three patients with recurrent PCNSL, there were 14 males and 9 females, and with a median age of 70 years old (from 65 to 82). All patients had diffuse large B-cell lymphoma, and the recurrence characteristics and previous treatment were shown in Table 1. The median KPS was 80 (range 60–90). The median time from initial PCNSL diagnosis to pemetrexed treatment was 11 months (range 4 to 25 months). All patients received at least two cycles treatment with pemetrexed, and the average duration of chemotherapy with pemetrexed was six cycles.

### 3.2. Response and Survival

After treatment, 10 patients survived except for 13 during the tumor procession among all patients. Among the ten survival cases, seven cases were alive until the end of the treatment, and three cases were alive until withdrawal from the treatment with unknown reason. Among the thirteen died cases, ten cases were dead during the tumor progression, and three cases were died including infection (2 patients) and unknown cardiac arrest (1 patients). Two patients died of respiratory failure after anti-infection treatment due to drug resistance. After the treatment, CR was achieved in 7 cases, PR in six cases, SD in four cases, and PD in six cases. According to the response for treatment, the overall response rate (CR + PR) was 56.5%, and the disease control rate (CR + PR + SD) was 73.9%. The median overall survival (OS) was 6.6 months (95% CI, 4.6–8.6), and the OS of recurrent PCNSL patients treated with pemetrexed is shown in Figure 1.

RETRACTED

### 3.3. Toxicities

Toxicities during the treatment are shown in Table 2. Myelosuppression, gastrointestinal reaction, and infection were the main adverse events during the treatment. The most severe adverse reaction was infection, which resulted in 3 deaths. Other common reactions included 9 cases of constipation and 8 cases of fatigue. There were 16 cases of leukopenia, anemia, and thrombocytopenia, including 11 cases of grade 1 and 2 and 5 cases of grade 3 and 4. After drug withdrawal or symptomatic treatment, the myelosuppression could be removed from the sixteen cases mentioned above. Nausea and vomiting were the common gastrointestinal reactions, including 7 patients of grade 1–2 and 2 patients of grade 3–4. In addition, 5-hydroxytryptamine-3 antagonist can relieve nausea and vomiting.

## 4. Discussion

PCNSL, as a rare variant of non-Hodgkin lymphoma, is an aggressive tumor confined to the central nervous system. Although extensive of efforts paid for exploring the treatment of PCNSL, patients still survive only a few months [6]. Unfortunately, nearly 50% of patients will relapse within 24 months of diagnosis, and about 50% of patients with recurrent PCNSL are older than 65 years. Currently, there is no general consensus on recurrent PCNSL in adolescent or the elderly. Due to profoundly influencing treatment choices in routine clinical practice, age has been recognized as an important prognostic factor for PCNSL. Radiation, such as whole brain radiotherapy, was considered to be inadequate for the elderly PCNSL patients due to the increased late neurotoxicity risk and shortly median survival time [16]. Methotrexate based high-dose chemotherapy is recognized as the standard treatment for PCNSL, and it has been reported that patients can tolerate methotrexate regimens and have good response rates [17–20]. However, some elderly patients cannot receive high-dose methotrexate due to impairment of renal function and other comorbidities. Pemetrexed, as an antitumor drug, is considered with advantage of recurrent PCNSL treatment compared with other chemotherapeutics. Several studies have reported that pemetrexed has better efficiency in the treatment of recurrent PCNSL [12–14]. Furthermore, the effectiveness of pemetrexed on recurrent PCNSL was also evaluated [14, 21]. However, these studies were only conducted to focus on general population. In our study, this is the first report focused on the elderly patients more than 65 years old to evaluate the efficacy of pemetrexed on recurrent PCNSL.

RETRACTED

A study evaluating the efficacy and safety of pemetrexed on elderly patients with initial PCNSL revealed that on the basis of the single-agent pemetrexed regimen (600 mg/m^2^), the overall response rate was 83.3% and the disease control rate with the median OS was 19.5 months [2]. In order to obtain a better prognosis, a higher dose of Jeffrey's (900 mg/m^2^) was chosen to increase central nervous system penetration in our study. Compared with initial elderly PCNSL, lower response rates and shorter survival time were associated with recurrent PCNSL in the elderly after the initial therapy with radiation or high-dose methotrexate. On the same of pemetrexed-based therapy, the disease control rate and the overall response rate in this study were 73.9% and 56.5%, respectively. The median OS was 6.6 months. Our results were expected.

Reducing toxicity in elderly recurrent PCNSL patients is a particular challenge. According to the dose of pemetrexed with 900 mg/m^2^, the toxicity in our patients was higher than reported in the previous studies treating with single-agent chemotherapy. In view of the toxicity, leukopenia, anemia, thrombocytopenia, nausea, vomiting, fatigue, and constipation were observed in this study. Two patients were died of grade 5 infection. Six patients experienced grade 4 adverse events, which including leukopenia (1 case), thrombocytopenia (1 case), vomiting (2 cases), fatigue (1 case), and constipation (1 case). There were 1 case with grade 3 anemia and 2 cases with grade 3 thrombocytopenia as well as fatigue and constipation. Most adverse events were controlled by corresponding treatment. The increased toxicity may be related to two main factors. One is the bodily harm from the initial PCNSL treatment and toxicity, and other one is a higher dose of pemetrexed which may directly increase toxicity risk.

The limitations of this study should be acknowledged. Firstly, due to collecting the data retrospectively, some patient selection bias might be introduced in this study. Secondly, the detailed patient characteristics such as comorbidities, trophic status, and geriatric assessments are not available. Last but not least, only the dose of 900 mg/m^2^ pemetrexed was considered in this study, and no comparison was made with the lower dose for more precise evaluation of efficacy and safety.

RETRACTED

## 5. Conclusion

This is the first study to evaluate the safety and efficacy of pemetrexed in the treatment of elderly patients with recurrent PCNSL. The results demonstrate that high-dose pemetrexed might be a feasible and effective treatment for recurrent PCNSL in the elderly, and clinical trials should be conducted to further confirm it.

## Figures and Tables

**Figure 1:** Overall survival of 23 recurrent elderly PCNSL patients treated with pemetrexed.

**Table 1:** Patients characteristics and therapy.

Patients	Age/gender	Position	KPS	Cycles	IT	Response	Outcome	PFS	OS
1	67/F	Primary recurrence	90	10	RT	CR	Alive	16.8+	16.8+
2	72/M	Ectopic recurrence	80	5	MTX	PR	Alive	10.2+	10.2+
3	78/M	Ectopic recurrence	80	8	MTX	PR	Death	9.2	10.3
4	82/F	Ectopic recurrence	80	4	RT	PR	Alive	8.8	10.1
5	65/F	Primary recurrence	90	3	MTX	CR	Alive	16.8+	16.8+
6	80/M	Primary recurrence	60	2	MTX	PD	Death	9.2	9.2
7	69/F	Ectopic recurrence	90	7	RT	CR	Alive	11.2+	11.2+
8	70/M	Ectopic recurrence	80	5	RT	PD	Death	9.5	9.5
9	70/M	Ectopic recurrence	80	9	MTX	CR	Alive	12.1	13.4+
10	65/F	Primary recurrence	80	11	MTX	CR	Death	7.2	9.1
11	74/M	Ectopic recurrence	90	4	MTX	PR	Death	6.2	7.8
12	76/F	Ectopic recurrence	80	8	MTX	SD	Death	2.4	2.8
13	68/F	Primary recurrence	60	7	RT	PD	Death	1.8	3.4
14	66/M	Primary recurrence	80	6	MTX	PD	Death	2.1	3.8
15	71/F	Primary recurrence	80	7	RT	PR	Alive	9.1	10.5
16	72/F	Ectopic recurrence	90	2	MTX	SD	Death	5.6	5.6
17	65/F	Primary recurrence	80	6	RT	CR	Alive	16.8+	16.8+
18	68/M	Primary recurrence	80	5	RT	SD	Death	3.4	6.1
19	75/F	Primary recurrence	60	5	MTX	PD	Death	6.6	6.6
20	69/F	Ectopic recurrence	80	7	MTX	SD	Death	4.2	5.8
21	70/F	Primary recurrence	80	9	MTX	CR	Alive	6.5	7.8+
22	77/M	Primary recurrence	60	8	RT	PD	Death	5.8	7.1
23	65/F	Metastasis	90	4	RT	SD	Alive	4.8	5.8

F, female; M, male; KPS, Karnofsky performance status; IT, initial treatment; RT, radiotherapy; MTX, methotrexate; CR, complete remission; PR, partial remission; SD, stable disease; PD, progressive disease; PFS, progression-free survival; OS, overall survival.

**Table 2:** Toxicities associated with pemetrexed.

Toxicities	Grade				
	1	2	3	4	5
Leukopenia	3	2	0	1	0
Anemia	2	0	1	0	0
Thrombocytopenia	2	2	2	1	0
ALT/AST	0	0	0	0	0
Infection	0	0	0	0	2
Vomiting	2	1	0	2	0
Nausea	3	1	0	0	0
Fatigue	3	2	2	1	0
Constipation	4	1	2	1	0

ALT, alanine aminotransferase; AST, aspartate aminotransferase.

## Data Availability

The datasets used and/or analyzed during the current study are available from the corresponding author on reasonable request.
